# TEGDMA (Triethylene Glycol Dimethacrylate) Induces Both Caspase-Dependent and Caspase-Independent Apoptotic Pathways in Pulp Cells

**DOI:** 10.3390/polym13050699

**Published:** 2021-02-25

**Authors:** Bálint Viktor Lovász, Gergely Berta, Edina Lempel, György Sétáló, Mónika Vecsernyés, József Szalma

**Affiliations:** 1 Department of Oral and Maxillofacial Surgery, University of Pécs, Medical School, 5. Dischka St., 7621 Pécs, Hungary; szalma.jozsef@pte.hu; 2 Department of Medical Biology and Central Electron Microscope Laboratory, University of Pécs Medical School, 12. Szigeti St., 7624 Pécs, Hungary; gergely.berta@aok.pte.hu (G.B.); gyorgy.setalo.jr@aok.pte.hu (G.S.J.); monika.hengl@aok.pte.hu (M.V.); 3 Szentágothai Research Centre, University of Pécs, Ifjúság Street 20, 7624 Pécs, Hungary; 4 Department of Restorative Dentistry, University of Pécs, Medical School, 5. Dischka St., 7621 Pécs, Hungary; lempel.edina@pte.hu

**Keywords:** TEGDMA, dental resin monomers, composite, apoptosis, caspase, composites

## Abstract

Monomers leached from resin-based composites (RBCs) may reach intrapulpal concentrations of the millimolar (mM) range, which could contribute to inflammation. The aim of this investigation was to assess the cytotoxicity of triethylene glycol dimethacrylate (TEGDMA) monomers on pulp cells as well as to identify molecular mechanisms leading to apoptosis. Pulp cells were harvested from molars extracted for orthodontic reasons and cultured through an explant method. To assess cytotoxicity, cells underwent a 5-day exposure to 0.75, 1.5, and 3 mM TEGDMA and were subject to cell counting and WST-1 staining. Based on the findings, cells were subsequently exposed to 0.1, 0.2, 0.75, 1.5, and 3 mM TEGDMA for 24 h to uncover the details of apoptosis. Changes in the production or cleavage of the apoptosis-specific proteins caspase-8, caspase-9, caspase-3, caspase-12, and Apoptosis-Inducing Factor (AIF) were measured by Western blot. The 5-day study showed concentration- and time-dependent cytotoxicity. Significant cell death was detected after 24 h with TEGDMA concentrations of 1.5 and 3 mM. One-day exposure to TEGDMA led to the activation of caspase-8, -9, -3, and -12 and an increased AIF production. Results suggest that relevant concentrations of TEGDMA monomers, leached from RBCs, induce apoptosis in pulp cells through both caspase-dependent as well as caspase-independent mechanisms. Endoplasmic reticulum stress and the activation of caspase-independent apoptotic pathways may be further mechanisms by which monomers induce apoptosis in pulp cells.

## 1. Introduction

Resin-based composite (RBC) is made up of soft resin matrix-containing methacrylates and dimethacrylates (e.g., bisphenol A-glycidyl methacrylate (BisGMA); urethane dimethacrylate (UDMA); triethylene glycol dimethacrylate (TEGDMA)), polymerized by an appropriate light source, that binds together hard inorganic filler particles, thereby ensuring adequate fluidity and plasticity for good handling and mechanical properties such as durability and longevity [1]. However, it has been observed in clinical practice that the application of resin-containing restorative materials in deep cavities can result in pulpal inflammation, which has been attributed to the monomer content [2]. Study of monomer toxicity has gained significant attention over the last decade. The conversion mechanism is not a chemically complete process. In general, 20–60% of the monomers stay unreacted, rarely exceeding 75% [1,3,4]. Various products undergo different degrees of conversion and, thus, produce different amounts of monomer extract [4,5], thereby leading to large variations in cytotoxicity [6]. Monomer products such as TEGDMA have been shown to be able to reach the pulp, with worst-case concentrations reported to be as high as 4 mM [7,8]. Although elution seems to be the highest in the first 24 h, it can continue for an extended period of time and may contribute to chronic pulpal inflammation [5,9].

Studies have shown TEGDMA cytotoxicity on various continuous cell lines as well as target cell isolates including human dental pulp cells [10,11,12]. Research into the mechanisms of TEGDMA monomer toxicity has so far uncovered DNA-damaging effects as well as its effects on cytokines, prostaglandin production, and metabolism [12,13,14,15]. Few studies have attempted to distinguish whether apoptosis or necrosis is the primary mechanism of cell death and only a handful of those investigated pulp cells [16]. Yeh et al. found apoptosis to be the primary mechanism of pulp cell death upon TEGDMA exposure [17]. Others have shown a concentration-dependent shift from apoptosis to necrosis [15,18,19]. While apoptosis is a controlled cell death without inflammation characterized by cell shrinkage, nuclear fragmentation, and formation of apoptotic bodies, necrosis is a result of massive cell damage leading to cell rupture and leakage of organelles. To date, research has shown that there are caspase-dependent and -independent apoptotic pathways. The former relies on the sequential activation of various proteolytic enzymes (caspases). The intrinsic pathway involves mitochondrial damage with a subsequent release of cytochrome c and activation of procaspase-9. The extrinsic pathway relies on signals originating from a death receptor activated by ligands such as the Fas ligand or Tumor Necrosis Factor-α (ΤΝF-α) and involves the activation of procaspase-8 with subsequent convergence with the intrinsic pathway on caspase-3 [20]. Another key organelle change implicated in apoptosis may be endoplasmic reticulum (ER) stress leading to caspase-12 translocation from the ER with subsequent activation of procaspase-9 and -3 [21]. Recent findings corroborate the existence of a caspase-independent apoptotic pathway also. Central to this mechanism is a mitochondrial polypeptide—Apoptosis-Inducing Factor (AIF)—causing chromatin condensation and DNA degradation [22].

Eliciting which apoptotic pathway leads to cell death would add valuable data to our understanding of monomer-induced pulpal toxicity. Two studies attempted to identify which caspase-dependent pathway mediates apoptosis in pulp cells. Yeh et al. detected the activation of the intrinsic pathway, while Batarseh et al. found evidence of both pathways mediating cell death [17,23]. To the best of the authors’ knowledge, no study has so far investigated the possible role of endoplasmic reticulum (ER) stress or the activation of caspase-independent apoptotic pathways in TEGDMA-induced pulp cell death.

In light of the abovementioned findings, the aim of this study is to confirm the dose-dependent cytotoxicity of TEGDMA monomers, and to confirm the predominant apoptotic pathway activated as well as determine whether ER stress and/or caspase-independent pathways are also induced in pulp cells by TEGDMA.

## 2. Materials and Methods

### 2.1. Reagents

All chemicals used were obtained from Sigma-Aldrich (now Merck KGaA, Darmstadt, Germany) unless stated otherwise.

### 2.2. Pulp Cell Culture

Pulp tissue was isolated from five healthy third molar teeth extracted for orthodontic reasons. The study was performed in accordance with the ethical standards laid down in the 1964 Declaration of Helsinki or comparable standards. All data were anonymized in line with patient confidentiality guidelines. Informed consent was obtained as per the protocol approved by the University of Pecs (Pecs, Hungary, under license No. PTE3026/2007). 

Following extraction, pulp tissue was isolated according to a technique described by Sun et al. [24] and cultured through an explant method in minimum essential medium eagle-alpha modification (Alpha MEM) containing ultraglutamine 1, ribonucleosides, and deoxyribonucleosides (Lonza, Basel, Switzerland) with the addition of 10% fetal bovine serum (FBS, Euroclone, Milan, Italy), and antibiotics (100 U/mL penicillin, 100 μg/mL streptomycin, 2.5 μg/mL amphotericin B). Culturing took place in a humidified atmosphere containing 5% CO_2_ at 37 °C. At 90% confluence, the passage to additional Petri dishes was undertaken. Cell cultures were first washed with phosphate-buffered saline (PBS, 1.37 mM NaCl, 0.27 mM KCl, 0.43 mM Na_2_HPO_4_·7H_2_O, 0.14 mM KH_2_PO_4_, pH 7.4) followed by trypsin (0.25% trypsin + 0.02% ethylene-diamine-tetraacetic acid (EDTA); Gibco, Grand Island, NY, USA) digestion for 10 min in a controlled, 37 °C, environment. Following two or three passages, cells were seeded at an arbitrary density of 2 × 10^4^ cells/cm^2^ based on previous experience with similar populations. Forty-eight hours hours prior to the start of the TEGDMA exposure, the medium was changed from 10% to 2% FBS-containing medium (without antibiotics) in order to decrease the potential signaling interference.

### 2.3. Monomer Exposure

In order to assess cytotoxicity, pulp cells were exposed to 0.75, 1.5, and 3 mM TEGDMA for a period of 5 days based on relevant literature data. Due to the kinetics of cell death observed in the 5-day study, for the investigations into the activation of various apoptotic pathways, cells were exposed to 0.1, 0.2, 0.75, 1.5, and 3 mM TEGDMA concentrations, however, this time for only 24 h.

### 2.4. Cell Counting

Following monomer exposure in 6-well plates, trypsin digestion was applied to collect the cells, followed by their suspension in Alpha MEM medium containing 10% FBS. One drop of the cell suspension was subsequently transferred into a counting chamber of a hemocytometer. Cells were counted using a phase contrast microscope, and cell numbers were calculated for each well.

For cell counting in marked fields of view, three areas were labeled on each well on the bottom of each culture plate. A phase contrast microscope was used to count the number of viable cells in the areas on days 1, 2, and 5 of the monomer exposure.

### 2.5. Fluorescence Microscopy

For illustrative purposes, nuclei were counterstained with Hoechst 33,342 (Calbiochem, La Jolla, CA, USA) to obtain representative images. Briefly, cells were rinsed with PBS at 37 °C, which was followed by 4% paraformaldehyde fixation at pH 7.4 and 4 °C for 4 h. Fixative was subsequently removed by further TBS washes (50 mM Tris-HCl, pH 7.4, 150 mM NaCl) and nuclei were counterstained with Hoechst 33,342 (Calbiochem, La Jolla, CA, USA). An Olympus FV-1000 laser scanning confocal system (Olympus Europa, Hamburg, Germany) with a 20× phase contrast dry objective was used to obtain the representative single optical slice images, which were merged with the pictures taken of the same viewing fields by the same phase contrast mode of the microscope.

### 2.6. WST-1 (Water-Soluble Tetrazolium Salts) Colorimetric Viability Assay

A WST-1 colorimetric assay, as an indicator of mitochondrial metabolism, was employed to demonstrate changes in viability. Following TEGDMA exposure, the medium was removed and 200 µL of WST- 1 reagent (Hoffmann-La Roche, Basel, Switzerland) in a 1:9 WST to 2% Alpha MEM medium ratio (180 µL of medium and 20 µL of WST dye) was added. Cells were subsequently stored at 37 °C for 4 h and then transferred to a 96-well plate. Absorbance was measured in 100 µL samples by a FluoStar Optima plate reader (BMG Labtech, Cary, NC, USA) at 440 nm.

### 2.7. Western Blotting

After TEGDMA treatment, cells were harvested and lysed as detailed in published studies [12]. Pulp cells were first collected in cold lysis buffer (50 mM Tris-base, pH 7.4, 10% glycerol, 150 mM NaCl, 1 mM EGTA, 1 mM Na-orthovanadate, 100 mM NaF, 5 μM ZnCl_2_, 10 μg/mL aprotinin, 1 μg/mL leupeptin, 1 mM PMSF, 1% Triton X-100), homogenized for 20 s, and then centrifuged for 30 min at 4 °C and at 40,000× *g*. Protein concentrations of the supernatants were measured (Lowry’s method, Detergent Compatible Protein Assay Kit, Bio-Rad, Hercules, CA, USA) and then diluted to contain an equal amount of 30 μg of protein. Following the addition of Laemmli buffer (prepared from 25 mL 1M Tris-HCl, pH 6.8, 40 mL glycerol, 8 g SDS, 10 mL 100 mM EGTA, 10 mL 100 mM EDTA, 1 mL 1% bromophenol blue; and distilled water to a total volume of 100 mL), samples were boiled for denaturation. Proteins were separated based on molecular size in a 10% SDS-containing polyacrylamide gel and then blotted to polyvinylidine fluoride (PVDF) membranes (Hybond-P, GE Healthcare, Little Chalfont, United Kingdom) by the Trans-Blot Turbo system (Bio-Rad, Hercules, CA, USA). Nonfat dry milk (3%) in TBS-Tween (10 mM Tris-base, 150 mM NaCl, 0.2% Tween-20, pH 8.0) was used to block nonspecific binding on the membrane. Rabbit polyclonal primary antibodies were added, specific to cleaved caspase-9, cleaved caspase-3, caspase-8, AIF (Cell Signaling Technology, Beverly, MA, USA), and caspase-12 (MBL International Corporation, Woburn, MA, USA), diluted to 1:1000 in the blocking solution, and then incubated overnight. Five washes with TBS-Tween were undertaken to remove excess antibodies. Incubation with a horseradish-peroxidase (HRP)-conjugated polyclonal goat anti-rabbit secondary antibody (Pierce, Thermo Fischer Scientific, Rockford, IL, USA) diluted to 1:10,000 in blocking solution followed. The enhanced chemiluminescent signal (Immobilon Western, Millipore Corporation, Billerica, MA, USA) was detected using a G:box gel documentation system (Syngene International Ltd., Bangalore, India). Membranes were then chemically stripped of antibodies (0.2M glycin-HCl, 0.2% Tween-20, 0.05%, pH 2.5) and reprobed using β-actin or GAPDH (Cell Signaling Technology, Beverly, MA, USA) rabbit polyclonal primary antisera as mentioned above to control the disparity in protein concentration among samples. Densitometry analysis was performed using the ImageJ software (National Institutes of Health, Bethesda, MD, USA).

### 2.8. Plotting of Experimental Data and Statistical Analysis

Data presented in the diagrams were gathered in a series of four independent experiments. Values shown are the means and standard deviations (± S.D.). The Kolmogorov–Smirnov test was used to test the normality of the distribution of the data. A one-way analysis of variance (ANOVA) test, supplemented with a Tukey’s post hoc test for multiple samples, was used to highlight the significance of differences. *P* values ˂ 0.05 were considered to be significant. Relevant significant differences are marked in the graphs and their corresponding P values are indicated in the figure legend.

## 3. Results

### 3.1. Cell Counting

Results of cell counting undertaken by two distinctive methods show a concentration- and time-dependent TEGDMA monomer toxicity on pulp cells. While significant cell death was detected at 24 h after exposure to 1.5 and 3 mM TEGDMA, 0.75 mM TEGDMA did not cause a significant increase in the number of dead cells (Figure 1, Figure 2, Figure 3 and Figure 4). Second- and fifth-day results showed the continued destruction of cells with near-complete cell death evident on the fifth day with exposure to 3 mM TEGDMA. Microscope images have been included to illustrate the changes in cell number over the course of the investigation.

### 3.2. WST-1 Colorimetric Viability Assay

Similar to the results of the above cell counting, WST-1 staining showed a significant reduction in cell viability at 24 h upon exposure to 1.5 and 3 mM TEGDMA. A concentration of 0.75 mM failed to decrease viability significantly at 24 h (Figure 5 and Figure 6). Second- and fifth-day readings confirmed the findings established by the above cell counting with minimal viability readings after 5 days of exposure to 1.5 and 3 mM TEGDMA. Based on the kinetics of cell death seen in the above results, it was decided that the treatment time applicable for the subsequent investigations would be 24 h.

### 3.3. Western Blotting

One-day exposure to TEGDMA led to an increase in the cleaved variants of all investigated caspases as well as to an induction of AIF production. Significant elevations in cleaved caspase-3, -8, and -9 were apparent after exposure to concentrations of 1.5 mM and 3 mM for caspase-3 (Figure 7), 0.1 and 0.2 mM for caspase-8, and 0.75, 1.5, and 3 mM in the case of caspase-9. The increase in caspase-12 (Figure 8) was determined to be significant above the concentration of 0.75 mM, while significant AIF production at 24 h occurred after exposure to 0.2 mM, 0.75 mM, and 1.5 mM TEGDMA (Figure 9).

## 4. Discussion

Since the observation that monomers from resin-based restorative materials may reach the pulp in the millimolar range and may be a cause of chronic pulp inflammation, an increasing number of studies have employed pulp cells in their toxicity investigations [2,7]. Although resin-based composites typically contain a mixture of monomers, the subject of this current study was chosen to be TEGDMA. Its hydrophilicity, surfactant, detergent-like properties, and low molecular weight render it capable of easily passing the cell membrane. Its relatively high proportion in modern composite formulations, 20–50%, makes TEGDMA a relevant target for RBC toxicity studies [8]. Pure TEGDMA has a concentration of 3.8 mol/L. Considering its relative content in RBCs and the postulated 500x dilution effect of 0.5 mm of dentine, the concentration applied herein was in the millimolar range, which is comparable to all recent cytotoxicity studies [25].

Results of the current investigation show a concentration- and time-dependent cytotoxicity for TEGDMA monomers on pulp cells over a period of 5 days. The number of viable cells decreased exponentially at all time-points upon exposures to 1.5 and 3 mM TEGDMA, with statistically significant deaths occurring already at 24 h. This is in line with the findings of Galler et al., who found 3 mM TEGDMA to reduce viability in pulp cells to 20% by 48 h while 0.3 and 1 mM TEGDMA only influenced viability minimally by the 96-h end-point of the study [12]. The viability assay employed within the framework of the current study confirmed the toxic concentration threshold to be somewhere between 0.75 and 1.5 mM. Similar threshold-values have been observed in earlier studies too on pulp cells, which found significant cell death to occur at 24 h above a concentration of 1 mM TEGDMA, which corresponded to a viability decrease of circa 20–30% [15,17,18]. However, toxic thresholds outside this range have also been reported. Two millimolar (2 mM) TEGDMA was the lowest concentration causing significant cell death in a study conducted by Paschalidis et al. Conversely, Batarseh et al. found significant cell death to take place already with exposure to 0.5 mM TEGDMA [23,26]. The former exclusively examined pulp stem cells, which are a subset of pulp cells. It is well documented that various cell populations have different sensitivities to TEGDMA [10,16]. As for the latter, although the principle of the lactate dehydrogenase (LDH) viability assay is the same as the WST-1 and MTT assays used in the current and aforementioned studies, respectively, the LDH test relies on the detection of different molecules and hence could have a slightly different sensitivity.

Mechanisms of TEGDMA toxicity may include an increase in reactive oxygen species (ROS) and cytokine production as well as the induction of oxidative DNA damage, DNA fragmentation, and micronuclei formation [27,28]. Recent studies have also focused on mapping out possible recovery mechanisms following exposure to sub-toxic concentrations of TEGDMA monomers. For instance, TEGDMA has been shown to induce the intrapulpal production of the anti-inflammatory molecule TGFβ-1 and various other growth factors such as FGF, PDGF, and VEGF, all of which play important roles in tissue repair and may contribute to pulp recovery [26]. Schneider et al. demonstrated an increase in cysteine uptake with a subsequent rise in intracellular glutathione formation as pulp cells were exposed to 0.3 mM TEGDMA [29].

The second finding of the present study was the confirmation of apoptosis as the mechanism of cell death as observed by the increase in apoptosis-specific caspases. The significance of findings pertaining to the pattern of pulp cell death lies in the lack of inflammation accompanying apoptosis as opposed to necrosis. Apoptosis has been demonstrated in a number of prior studies and among other things was found to correlate with the inhibition of PI3K signaling [18]. Chang et al. detected a decrease in the expression of cdc2, cyclin B1, and cdc25C in pulp cells upon exposure to low toxic TEGDMA concentrations, leading to S phase arrest and a concurrent rise in the number of apoptotic cells [15]. Implicating NADPH oxidase 4 as a possible inducer of apoptosis in pulp cells, Yeh et al. found that silencing the expression of the above enzyme resulted in a steep decline in ROS production and almost completely abolished TEGDMA-induced apoptosis [17].

In a bid to specify which apoptotic pathway is employed, Batarseh et al. used an antibody array to detect changes in the levels of various apoptosis-specific proteins. Bid, Bim, cytochrome c, caspase-8, and caspase-3 were found to increase in pulp cells upon exposure to low concentrations of TEGDMA, implying that both intrinsic and extrinsic pathways had been activated [23]. Contrastingly, Yeh et al. observed a rise only in caspase-9 cleavage, thus suggesting the intrinsic pathway to mediate TEGDMA-induced cell death [17]. In accordance with the first author, the current study has also found both pathways to be activated. TEGDMA exposure led to a significant rise in cleaved caspase-8 as well as cleaved caspase-9 and caspase-3 levels. Multiple studies have confirmed the induction of ROS production to be one of the main mechanisms of monomer toxicity [13,17,29]. ROS in turn has been shown to play a role in the activation of both intrinsic and extrinsic caspase-dependent apoptotic pathways [20]. In addition, TEGDMA exposure has also been demonstrated to lead to a significant rise in TNF-α expression in pulp cells, which could provide a mechanism for the initiation of the extrinsic pathway [23]. A decline in anti-apoptotic protein BCL-xL leading to mitochondrial depolarization and cytochrome release, as observed in pulp cells in connection with TEGDMA exposure, supports the activation of the intrinsic pathway [20].

To the best of the authors’ knowledge alternative apoptotic pathways have not yet been investigated in connection with TEGDMA exposure. Additional to the aforementioned findings, the present study demonstrated a rise in AIF and cleaved caspase-12 levels in pulp cells upon exposure to TEGDMA monomers. A recent development has been the identification of endoplasmic reticulum (ER) stress as a further possible initiator of apoptosis through the release of caspase-12. The ER is principally responsible for post-translational modification of proteins and oxidative protein folding (OPF). These processes rely on a tightly regulated intraluminal redox homeostasis ensured, among other things, by a very specific intraluminal ratio of glutathione (GSH) to reduced glutathione (GSSG). Although the oxidative environment favors OPF, excessive ROS production and GSH depletion, both of which have been shown to be an effect of TEGDMA exposure, can lead to the destruction of this redox balance [30]. As a primary site of tertiary and quaternary folding of proteins, this leads to the formation of unfolded protein aggregates, which in turn activates, through diverse signaling mechanisms, membrane-bound caspase-12. Translocation of caspase-12 from the ER membrane leads to procaspase-9 activation and convergence with other pathways on caspase-3 [21]. AIF is a mitochondrial protein residing in the intermembranous space with both resident housekeeping and possible apoptosis effector functions. Redox energy crisis may lead to mitochondrial permeabilization. Upon release, AIF translocates to the nucleus and induces large-scale DNA fragmentation to 20 kb and 50 kb fragments and subsequent condensation in a caspase-independent way, thereby leading to cell death [22]. The present findings of increased levels of AIF and caspase-12 have furthered our understanding of monomer toxicity.

Limitations of the current study may include the in vitro nature of the investigation. The present study demonstrated significant cytotoxicity in controlled conditions. Many additional factors may influence intrapulpal monomer concentration and toxicity in vivo, such as circulation, pressure, outward dentinal fluid flow, as well as chemical interactions with dentine. Pulp cells were obtained from healthy teeth extracted for orthodontic reasons. Composite restorations are placed in destructed teeth. Stressed pulp cells may respond slightly differently to monomer exposure. Additionally, in the present study cells were exposed to TEGDMA only. As commercially available composite mixtures contain various other monomers, combinatorial studies would be useful to elicit possible synergistic effects that would apply better to the in vivo situation and are among the future plans for the research group.

## 5. Conclusions

In conclusion, the current in-vitro study has confirmed the concentration- and time- dependent cytotoxicity of TEGDMA monomers on pulp cells. Both intrinsic and extrinsic apoptotic pathways were found to be activated by the monomers. ER stress and AIF may be novel mediators of monomer-induced cell death.

## Figures and Tables

**Figure 1:** Number of viable pulp cells at various time-points of the 5-day exposure to 0.75, 1.5, and 3 mM triethylene glycol dimethacrylate (TEGDMA), as measured by a hemocytometer (sample number: *n* = 2).

**Figure 2:** Number of viable pulp cells at various time-points of the 5-day exposure to 0.75, 1.5, and 3 mM TEGDMA, as counted in marked fields of view (sample number: *n* = 2).

**Figure 3:** Number of viable pulp cells at various time-points of the 5-day exposure to 0.75, 1.5, and 3 mM TEGDMA, as measured by a hemocytometer and counted in marked fields of view. The hemocytometer graph presents the absolute number of viable cells, while the marked fields of view graph plots the decrease in the number of viable cells as a ratio relative to the control cell number at the start of the experiment. * = significantly different from the untreated control of the first day (for the hemocytometer, *P* = 0.0018, *P* = 0.0002 at 1.5 mM and 3 mM TEGDMA concentrations, and *P* = 0.0293, *P* = 0.0004 at 1.5 mM and 3 mM TEGDMA concentrations for the viewing field data, respectively, sample number: *n* = 2).

**Figure 4:** Illustrative microscope images showing the change in viable cell number over the course of the investigation (sample number: *n* = 2, 20X dry objective, scale bar represents 100 µm).

**Figure 5:** Viability changes in pulp cells over the course of the 5-day exposure to 0.75, 1.5, and 3 mM TEGDMA as detected by the Water-Soluble Tetrazolium-1 assay (sample number: *n* = 3).

**Figure 6:** Viability changes in pulp cells over the course of the 5-day exposure to 0.75, 1.5, and 3 mM TEGDMA as detected by the Water-Soluble Tetrazolium-1 assay. The graph depicts viability values as a ratio relative to the untreated cells at the start of the experiment. * = significantly different from the 1st day untreated control (*P* = 0.0293, 0.0004 for 1.5 mM and 3 mM, respectively, sample number: *n* = 3).

**Figure 7:** Immunoblots showing the changes in the levels of cleaved caspase-3, -8, and -9 in pulp cells after a 1-day exposure to 0.1, 0.2, 0.75, 1.5, and 3 mM TEGDMA. GAPDH or β-actin bands, obtained by reprobing the Western blot membrane, served as a loading control each time. Results of the quantitative analysis of densitometry data are illustrated below each blot (gathered by ImageJ). * = significantly different from the untreated control (in the case of the cleaved caspase-3 *P* = 0.0174 and *P* < 0.0001 at 1.5 mM and 3 mM, respectively; for the uncleaved caspase-8 *P* = 0.0002, P< 0.0001, P< 0.0001, and P< 0.0001 at 0.2 mM, 0.75 mM, 1.5 mM, and 3 mM, respectively; for the cleaved caspase-8 *P* = 0.0002, *P* < 0.0001, *P* < 0.0001, and *P* < 0.0001 at 0.2 mM, 0.75 mM, 1.5 mM, and 3 mM, respectively; in the case of the cleaved caspase-9 *P* = 0.0208, *P* < 0.0001, *P* < 0.0001, *P* < 0.0001, and *P* = 0.0035 at 0.1 mM, 0.2 mM, 0.75 mM, 1.5 mM, and 3 mM, respectively, sample number: *n* = 3).

**Figure 8:** Immunoblots showing the changes in the levels of cleaved caspase-12 after a 1-day exposure to 0.1, 0.2, 0.75, 1.5, and 3 mM TEGDMA. β-actin bands, obtained by reprobing the Western blot membrane, served as a loading control each time. Results of the quantitative analysis of densitometry data are illustrated below the blot. * = significantly different from the untreated control (*P* = 0.0074, *P* < 0.0001, and *P* < 0.0001 at 0.75 mM, 1.5 mM, and 3 mM, respectively, sample number: *n* = 3).

**Figure 9:** Western blots representing the alterations in Apoptosis-Inducing Factor (AIF) concentrations after a 1-day exposure to 0.1, 0.2, 0.75, 1.5, and 3 mM TEGDMA. β-actin is presented as a means of loading control. Results of the quantitative analysis of densitometry data are illustrated below the blot. * = significantly different from the untreated control (*P* < 0.0001, *P* = 0.0074, and *P* = 0.0158 at 0.2 mM, 0.75 mM, and 1.5 mM respectively, sample number: *n* = 3).

## Data Availability

The data presented in this study are available on request from the corresponding author.
